RETRACTED

# CUL4B promotes bladder cancer metastasis and induces epithelial-to-mesenchymal transition by activating the Wnt/β-catenin signaling pathway

**DOI:** 10.18632/oncotarget.20455

**Published:** 2017-08-24

**Authors:** Xia-Wa Mao, Jia-Quan Xiao, Gang Xu, Zhong-Yi Li, Hui-Feng Wu, Yi Li, Yi-Chun Zheng, Nan Zhang

**Affiliations:** ^1^ Department of Urology, The Second Affiliated Hospital of Zhejiang University School of Medicine, Hangzhou 310009, P.R. China

**Keywords:** CUL4B, Wnt/β-catenin signaling pathway, bladder cancer, epithelial-to-mesenchymal transition, proliferation

## Abstract

Increased expression of cullin 4B (CUL4B) is linked to progression in several cancers. This study aims to explore the effects of CUL4B on bladder cancer (BC) metastasis and epithelial-to-mesenchymal transition (EMT) and potential correlation to the Wnt/β-catenin signaling pathway. We collected BC tissues and adjacent normal tissues from 124 BC patients. Quantitative real-time polymerase chain reaction (qRT-PCR) and western blotting were employed in order to detect the expression of Wnt/β-catenin signaling pathway-related proteins and EMT markers. MTT and Transwell assays were used in order to measure cell proliferation, migration, and invasion. BC 5637 cells were transfected with control, siRNA scramble control (siRNA-NC), si-CUL4B, and CUL4B or Wnt inhibitory factor 1 (WIF-1) overexpression constructs. Levels of CUL4B mRNA and protein were increased in BC tissues in comparison with the adjacent normal tissues. CUL4B expression was negatively correlated with the expression of E-cadherin and positively correlated to the expression of N-cadherin and Vimentin. Compared to the control group, levels of β-catenin, cyclinD1, c-myc, MMP7, and EMT markers were reduced, whereas phosphorylated GSK3β^Ser9^ and E-cadherin levels were increased in the si-CUL4B and WIF-1 groups. In addition, cell proliferation, migration, and invasion abilities were also increased. Increasing CUL4B expression had the opposite effect. These findings suggest that CUL4B induces EMT and promotes metastasis of BC by activating the Wnt/β-catenin signaling pathway.

## INTRODUCTION

Bladder cancer (BC) is characterized by its high recurrence and mortality rate, and is one of the most prevalent genitourinary malignancies [1, 2]. Each year more than 350,000 patients are diagnosed with BC around the world, with more than 70,000 cases in the United States alone [3]. A majority of diagnosed BCs are non-invasive early stage tumors, but BC accounts for one-third of non-muscular invasive diseases which eventually metastasize and progress to a myometrial invading disease [4, 5]. Factors that affect the overall mortality rate of BC include age, smoking history, chemical exposure (including aniline dyes and aromatic amines), and contact with carcinogens [3, 6]. Neoadjuvant cisplatin-based chemotherapy in combination with radical cystectomy is the recommended treatment strategy for advanced stage BC [7, 8], but there is a need for more effective therapy methods. The search for new therapeutic treatments is dependent on the identification of the molecular mechanisms of BC progression, which should reveal potential new targets [9].

RETRACTED

The CUL4B gene, located on the X chromosome, has been implicated in X-linked intellectual disability [10] and encodes a protein primarily localized to the nucleus. The expression of CUL4B is upregulated in lung and colorectal cancer [11–13]. CUL4B expression is closely associated with the invasion, differentiation, and metastasis of colon cancer cells [13]. CUL4B also promotes cell proliferation and inhibits cell apoptosis in patients with osteosarcoma [14]. The Wnt/β-catenin signaling pathway can affect gene expression and cell migration [15]. β-catenin is of great importance to signal transduction and protein stability, and is enriched locally under the influence of the Wnt signaling pathway [16]. In addition, immunosuppressive cells, such as regulatory T cells and myeloid derived suppressor cells (MDSCs), and β-catenin inhibit the Wnt pathway's function [17, 18]. The Wnt/β-catenin signaling pathway plays a crucial role in driving EMT and metastasis [19], but the mechanism behind the Wnt/β-catenin signaling pathway regulation in EMT is still unclear [20]. EMT refers to the process by which tumor cells transform from polar epithelial-like cells into free moving interstitial cells with increased potential for migration and invasion [21]. EMT is important in cancer progression, as it damages the integrity of the epithelium and promotes metastasis [22]. Numerous signaling pathways, such as the TGF-β and Notch signaling pathways, are involved in the EMT process [23]. We speculated that the Wnt/β-catenin signaling pathway activates EMT in BC and targets CUL4B to promote metastasis. This study aims to elucidate the molecular mechanisms that promote the invasion and metastasis of BC cells by measuring the expression of CUL4B, EMT markers (E-cadherin, N-cadherin, and Vimentin), and Wnt/β-catenin signaling pathway-related proteins.

## RESULTS

### Expression levels of CUL4B and EMT markers in the BC and adjacent normal tissues

Immunohistochemistry (IHC) showed that CUL4B was predominantly found in the nucleus, E-cadherin was found in the cell membrane, and N-cadherin and Vimentin were found in the cytoplasm (Figure 1A). Patients (n = 59) exhibited a high expression of CUL4B in the adjacent normal tissues (59/142), and 87 exhibited a high expression of CUL4B in the BC tissues (87/142) (χ^2^ = 11.05, *P* = 0.01). High E-cadherin expression was observed in BC tissues of 30.3% patients (43/142) and in adjacent normal tissues of 56.3% patients (80/142) (χ^2^ = 19.63, *P* < 0.001). N-cadherin was highly expressed in the BC tissues of 47.9% patients (68/142) and in adjacent normal tissues of 11.3% patients (16/142) (χ^2^ = 14.71, *P* < 0.001). Vimentin expression was high in BC tissues of 19.0% patients (27/142) whereas a high expression was observed in adjacent normal tissues of only 7.0% patients (10/142) (χ^2^ = 8.98, *P* = 0.003) (Figure 1B).

RETRACTED

**Figure 1:** Expression of CUL4B and EMT marker proteins in BC tissues and adjacent normal tissues **(A)** Expression of CUL4B and EMT markers detected by IHC. The percentage of cells expressing CUL4B, E-cadherin, N-cadherin, and Vimentin in the adjacent normal tissues was 2%, 87%, 5%, and 3%, respectively; the staining intensity was 0, 3, 0, and 0, respectively. The percentage of cells expressing CUL4B, E-cadherin, N-cadherin and Vimentin in the BC tissues was 28%, 16%, 70%, and 3%, respectively. The staining intensity was 3, 1, 3, and 3, respectively; **(B)** the percentage of high expression of CUL4B and EMT marker proteins.

### CUL4B protein level correlates with clinicopathological characteristics of advanced BC

Patients exhibiting a high CUL4B protein expression were generally in TNM stage III-IV (*P* = 0.015) with lymph node metastasis (N2-N3) (*P* = 0.005) and muscle invasion (T3-T4) (*P* = 0.001). Furthermore, the level of CUL4B protein expression was not correlated to the gender or age of the patients (all *P* > 0.05) (Table 1).

**Table 1:** The relations between CUL4B and clinicopathologic characteristics of BC patients

Influence factor	Case	CUL4B		*P*
		High expression	Low expression	
Age				0.601
< 65	83	49	34	
≧ 65	59	38	21	
Gender				0.69
Male	107	67	40	
Female	35	20	15	
TNM Stage				0.015
I-II	59	29	30	
III-IV	83	58	25	
Lymph node metastasis				0.005
N0-N1	58	27	31	
N2-N3	84	60	24	
Myometrial invasion				0.001
T1-T2	75	36	39	
T3-T4	67	51	16	

TNM, tumor-node-metastasis; BC, bladder cancer.

### Association between the expression levels of CUL4B and EMT markers in BC tissues

Spearman's correlation showed that the expression of CUL4B protein in BC tissues was negatively correlated with E-cadherin (r = –0.462, *P* < 0.001) but positively correlated to N-cadherin expression (r = 0.318, *P* < 0.001) and Vimentin expression (r = 0.201, *P* = 0.016) (Table 2).

**Table 2:** The correlation of CUL4B with EMT markers in bladder cancer tissues and adjacent normal tissues

EMT markers	CUL4B		*r*	*P*
	High expression	Low expression		
E-cadherin				
High expression	17	36	–0.462	< 0.001
Low expression	0	19		
N-cadherin				
High expression	68	26		
Low expression	19	29	0.318	< 0.001
Vimentin				
High expression	22	5		
Low expression	65	50	0.201	0.016

EMT, epithelial-to-mesenchymal transition; BC, bladder cancer.

RETRACTED

### Expression levels of CUL4B and EMT markers in BC cell lines EJ, 5637, T24, and RT-4

QRT-PCR was employed in order to measure the mRNA expression of CUL4B and EMT markers in BC cell lines EJ, 5637, T24, and RT-4. CUL4B, N-cadherin, and Vimentin mRNA levels were lowest in EJ cells and highest in 5637 cells. E-cadherin mRNA level was highest in EJ cells and lowest in 5637 cells. Furthermore, CUL4B, E-cadherin, N-cadherin, and Vimentin mRNA levels were expressed at intermediate levels in T24 and RT-4 cells. Western blotting confirmed that protein expression in BC cell lines was consistent with the mRNA expression (Figure 2). The expression of CUL4B was evidently highest in 5637 cells and lowest in EJ cells. Therefore, 5637 cells were chosen for subsequent experiments.

**Figure 2:** The mRNA and protein expression in BC cell lines EJ, 5637, T24, and RT-4 **(A)** CUL4B, E-cadherin, N-cadherin, and Vimentin mRNA expression; **(B)** CUL4B, E-cadherin, N-cadherin and Vimentin protein expression; **(C)** cartogram of CUL4B, E-cadherin, N-cadherin, and Vimentin protein expression. * compared with cell line 5637, *P* < 0.05.

### siRNA and overexpression constructs altered CUL4B mRNA levels

Figure 3A shows the relative mRNA expression of CUL4B in 5637 cells in the si-CUL4B group was lower than the siRNA-NC and control groups (all *P* < 0.05). The CUL4B and CUL4B + WIF-1 groups exhibited higher CUL4B mRNA expression than the siRNA-NC and control groups (all *P* < 0.05). No significant CUL4B mRNA expression differences were found among the siRNA-NC, WIF-1, and control groups (*P* > 0.05). Furthermore, CUL4B siRNA reduced CUL4B by 63%. Western blotting confirmed that the changes in protein levels were consistent with the RNA levels (Figure 3B and 3C).

**Figure 3:** Relative mRNA and protein expression of CUL4B in each group **(A)** Relative mRNA expression of CUL4B in each group detected by qRT-PCR; **(B)** protein expression of CUL4B detected by western blotting; **(C)** relative CUL4B protein expression in each group. * compared with the control group, *P* < 0.05.

### Effect of CUL4B on the Wnt/β-catenin signaling pathway

si-CUL4B and WIF-1 treatment of 5637 cells significantly reduced mRNA and protein levels of the Wnt/β-catenin signaling pathway components β-catenin, cyclinD1, c-myc, and MMP7 and increased the level of phosphorylated GSK3β^Ser9^ (p-GSK3β^Ser9^) (all *P* < 0.05). Exogenous expression of CUL4B increased mRNA and protein levels of β-catenin, cyclinD1, c-myc, and MMP7 and decreased the amount of p-GSK3β^Ser9^ (all *P* < 0.05). There were no significant p-GSK3β^Ser9^ protein expression differences among the siRNA-NC, CUL4B + WIF-1, and control groups (all *P* > 0.05). In addition, no GSK3β mRNA expression differences were found in any group (*P* > 0.05) (Figure 4). These findings indicate that CUL4B activates the Wnt/β-catenin signaling pathway, and si-CUL4B suppresses the Wnt/β-catenin signaling pathway.

RETRACTED

**Figure 4:** Effect of CUL4B on the Wnt/β-catenin signaling pathway **(A)** mRNA expression of β-catenin, cyclinD1, c-myc, and MMP7 in each group determined by qRT-PCR; **(B)** expression of β-catenin/β-actin, cyclinD1/β-actin, c-myc/β-actin, and MMP7/β-actin in each group determined by western blotting; **(C)** cartogram of protein expression of β-catenin, cyclinD1, c-myc and MMP7 in each group; **(D)** mRNA expression of GSK3β in each group determined by qRT-PCR; **(E)** expression of t-GSK3β/GAPDH, p-GSK3β^Ser9^/GAPDH in each group determined by western blotting; **(F)** cartogram of levels of p-GSK3β^Ser9^/t-GSK3β in each group. * compared with the control group, *P* < 0.05.

### CUL4B promotes EMT *in vitro*

Figure 5 shows that si-CUL4B and WIF-1 increased E-cadherin mRNA and protein levels, and decreased N-cadherin, Vimentin, ZEB1, ZEB2, and Snail1 mRNA and protein levels in comparison to the control group (all *P* < 0.05). Increased expression of CUL4B resulted in opposite trends, and there was no difference among the CUL4B + WIF-1 and siRNA-NC group (*P* > 0.05). These findings suggest that transfection with CUL4B siRNA reverses the downregulation of E-cadherin and upregulation of ZEB1, ZEB2, Snail1, N-cadherin, and Vimentin that occur in EMT.

**Figure 5:** Effect of CUL4B on EMT *in vitro* **(A)** mRNA expression of E-cadherin, N-cadherin, Vimentin, Snail1, ZEB1, and ZEB2 in each group detected by qRT-PCR; **(B)** protein expression of E-cadherin, N-cadherin, Vimentin, Snail1, ZEB1, ZEB2, and GAPDH in each group detected by western blotting; **(C)** cartogram of protein expression of E-cadherin, N-cadherin, Vimentin, Snail1, ZEB1, and ZEB2 in each group. * compared with the control group, *P* < 0.05.

### CUL4B increases proliferation of BC 5637 cells *in vitro*

MTT assay (Figure 6) showed that cell viability was elevated in all three groups at each time period. Cell proliferation in the si-CUL4B and WIF-1 group was lower than the control group (all *P* < 0.05). CUL4B overexpression promoted cell proliferation in the CUL4B group (*P* < 0.05). No significant cell proliferation differences were found among the siRNA-NC, CUL4B + WIF-1, and control groups (all *P* > 0.05).

RETRACTED

**Figure 6:** Effect of CUL4B on BC cell proliferation * compared with the control group, *P* < 0.05.

### CUL4B increases the migration and invasion of BC 5637 cells *in vitro*

The Transwell assay (Figure 7) showed that si-CUL4B and WIF-1 inhibited the migration and invasion abilities of BC cells in comparison to the control group (all *P* < 0.05). Increased CUL4B expression amplified the migration and invasion abilities of BC cells (all *P* < 0.05). No migration and invasion ability differences were observed among the siRNA-NC, CUL4B + WIF-1, and control groups (all *P* > 0.05).

**Figure 7:** Effect of CUL4B on BC cell migration and invasion **(A)** CUL4B interference inhibited the cell migration ability in each group detected by Transwell assay; **(B)** the number of migrating cells in each group; **(C)** CUL4B interference inhibited the cell invasion ability in each group detected by Transwell assay; **(D)** the number of invasive cells in each group. * compared with the control group, *P* < 0.05.

### CUL4B increases tumor growth *in vivo*

A subcutaneous xenograft BC tumor model was established in BALB/c nude mice in order to verify the effects of CUL4B on tumor growth. At the 10^th^ day after inoculation, the tumor volume in the si-CUL4B group was reduced in comparison to the siRNA-NC and control groups (all *P* < 0.05), the tumor volume in the CUL4B group was larger than the control group (*P* < 0.05), and no tumor volume differences were found among the siRNA-NC and control groups (all *P* > 0.05) (Figure 8A). Compared to the control group, the tumor weight in the si-CUL4B group was lower (all *P* < 0.05), the tumor weight in the CUL4B group was higher (*P* < 0.05), and there was no difference in tumor weight among the siRNA-NC and control groups (all *P* > 0.05) (Figure 8B).

**Figure 8:** Effect of CUL4B on tumor growth in nude mice *in vivo* **(A)** Tumor volume in each group; **(B)** tumor weight in each group. * compared with the control group, *P* < 0.05.

### CUL4B promotes EMT *in vivo*

Results of qRT-PCR and IHC show that E-cadherin mRNA and protein expression was elevated and N-cadherin and Vimentin expression was decreased in the si-CUL4B group in comparison to the control group (all *P* < 0.05). The expression of CUL4B and EMT markers in the CUL4B group followed opposite trends (all *P* < 0.05). In addition, there were no significant mRNA and protein expression of E-cadherin, N-cadherin, and Vimentin differences among the siRNA-NC and control group (all *P* > 0.05) (Figure 9).

RETRACTED

**Figure 9:** Effect of CUL4B on EMT *in vivo* **(A)** mRNA expression of E-cadherin, N-cadherin, and Vimentin in nude mouse xenografts determined by qRT-PCR; **(B)** the protein expression of E-cadherin, N-cadherin, and Vimentin in nude mouse xenografts detected by IHC. * compared with the control group, *P* < 0.05.

### CUL4B increases lung metastasis in nude mice

The number of metastatic lung nodules of mice was significantly reduced in the si-CUL4B group in comparison to the control group (*P* < 0.05), while the number was evidently increased in the CUL4B group (*P* < 0.05). BC cells were enriched in lung areas of mice in the siRNA-NC and control group (Figure 10).

**Figure 10:** Effect of CUL4B on the number of lung metastases in BC cells in each group * compared with the control group, *P* < 0.05.

## DISCUSSION

The current study was conducted in order to explore the expression of CUL4B, EMT markers (E-cadherin, N-cadherin, and Vimentin) and the Wnt/β-catenin signaling pathway-related proteins in BC tissues to elucidate the role of CUL4B in promoting the invasion and metastasis of BC.

CUL4B is a part of the Cullin4B-Ring E3 ligase complex (CRL4B) and is highly expressed in various cancer types such as colorectal cancer [12]. In addition, CUL4B is involved in a series of controlled processes related to cancer initiation [14]. High CUL4A expression was found in breast and colon cancers, and CUL4A together with other several cyclin-dependent kinase inhibitors targets p53 in cultured cells [13, 24]. This is consistent with our findings that CUL4B expression is elevated in BC tissues compared to adjacent normal tissues. In a previous study, knockdown of CUL4B inhibited cell proliferation in colorectal cancer by suppressing the Wnt/β-catenin signaling pathway [12]. Incidentally, it is hypothesized that CUL4B activates the Wnt/β-catenin signaling pathway by protecting β-catenin from GSK3-mediated degradation and CUL4B-mediated epigenetic silencing of Wnt signaling pathway antagonists.

Downregulation of CUL4B decreased mRNA and protein expression of β-catenin and cyclinD1. This suggests that siRNA acting against CUL4B inhibits the expression of proteins related to the Wnt/β-catenin signaling pathway. A previous study found that Wnt antagonist expression is repressed by CRL4B–PRC2 upon CUL4B upregulation, which in turn promotes Wnt/β-catenin signaling pathway activity and drives tumorigenesis [25]. Furthermore, Cheng et al. proved that CUL4B and β-catenin expression is upregulated in liver tumors, and that CUL4B increased the expression of β-catenin *in vitro* [26].

EMT is regarded as a critical step in tumor metastasis and invasion. The results of our study indicated that CUL4B knockdown using siRNA upregulated the expression of E-cadherin and downregulated the expression of N-cadherin, Vimentin, ZEB1, ZEB2, and Snail1, suggesting that CUL4B driven tumor proliferation, migration, and invasion. Interestingly, E-cadherin is not normally expressed in prostate cancer, but all cancer cells exhibited positive expression of N-cadherin and Vimentin [27]. In regard to epithelial cells, the reduced expression of E-cadherin and increased expression of N-cadherin and Vimentin indicates tumor advancement to a metastatic phenotype [28]. It is reported that CUL4B knockdown in non-small cell lung cancer cells (NSCLC) inhibits the progression of EMT and reduces the expression of β-catenin, cyclin D1, and c-Myc in NSCLC [11]. Moreover, in a recently created mouse model, overexpression of CUL4B greatly promoted the proliferation of hepatocytes in liver cells [29]. As a member of the seven cullin proteins, CUL7 plays a key role in the regulation of EMT of the trophoblast cell lineage. CUL7 expression is accompanied by a complete loss of E-cadherin and an elevation of the two mesenchymal markers, Vimentin and N-cadherin [30]. It is suggested that knockdown of CUL4B significantly decreases cell proliferation and colony formation, causing the arrest of G1 phase cell cycle through downregulation of cyclin D1 and upregulation of p16 [31]. Considering the indispensable role of EMT in promoting the progression of various carcinomas, and the fact that BC invasion shares many similarities with the invasion of other tumor cells, our results raise the interesting hypothesis that CUL4B interference can inhibit the activation of the Wnt/β-catenin signaling pathway and suppress EMT and metastasis in BC.

RETRACTED

In summary, our study revealed that CUL4B induces EMT, activates the Wnt/β-catenin signaling pathway, and promotes proliferation, migration, and invasion of BC cells. Our study also suggests a possible pathological mechanism of metastasis and progression in BC. Therefore, CUL4B may represent a novel therapeutic target for BC treatment. The inhibitory effect of siRNA gradually diminishes with cell proliferation. Therefore, we plan to monitor the effect of CUL4B knockdown on tumor size in nude mice tumor size at different time periods in future studies. Additionally, possible regulators of CUL4B that promote EMT of BC cells should be investigated further.

## MATERIALS AND METHODS

### Ethics statement

This study was conducted based on the protocols proposed by the ethics committee of the Second Affiliated Hospital of Zhejiang University School of Medicine. Informed written consents were obtained from all patients participating in the study. The animal experiment was carried out in strict accordance with the recommendations in the Guide for the Care and Use of Laboratory Animals of the National Institutes of Health. All efforts were made to minimize animal suffering along the experiment.

RETRACTED

### Study subjects

BC tissues were collected from 142 patients (107 males, 35 females; age, 32-68 years; calculated mean age 56.4 ± 10.2 years) with primary transitional cell carcinoma of the bladder who underwent surgical resection from January 2012 to January 2015 in the Second Affiliated Hospital of Zhejiang University School of Medicine. No patients included in the study underwent radiotherapy, chemotherapy, or hormone therapy and no patients were suffering from other acute or chronic diseases or malignant tumors. TNM staging was determined in accordance with the criteria of the American Joint Cancer Committee (AJCC) [32]. Accordingly, there were 59 patients in stage I and II, 83 patients in stage III and IV. In addition, there were 58 patients with lymph node metastasis (N0-N1), 84 patients with N2-N3, 75 cases of muscle-invasive BC (T1-T2), and 67 cases of T3-T4. Adjacent normal tissues were collected as the control group. After washing with normal saline, a portion of each sample was cryopreserved in liquid nitrogen. Another portion of each sample was fixed with neutral buffered formalin for 24 h, and embedded in paraffin for further experimentation.

### IHC

Paraffin-embedded specimens (BC tissues, adjacent normal tissues, and tumor tissues from nude mice) were sliced into 4 μm thick serial sections and placed in an incubator at 70°C for 15 min. The specimens were dehydrated using gradient ethanol and present endogenous peroxidases were inactivated using H_2_O_2_. The dehydrated specimens were rinsed in phosphate buffered saline (PBS) three times (each time for 5 min) and incubated in normal goat serum for 15 min at room temperature. Subsequently, primary antibodies were diluted using 20-30 μl PBS: CUL4B (ab211118, diluted at a ratio of 1: 100; Abcam, Inc., Cambridge, Massachusetts, USA), E-cadherin (#3195; diluted at a ratio of 1: 100; Cell Signaling Technologies (CST), Beverly, Massachusetts, USA), N-cadherin (#8480; diluted at a ratio of 1: 100; CST, Beverly, Massachusetts, USA), and Vimentin (#5741; diluted at a ratio of 1: 100; CST, Beverly, Massachusetts, USA). After dilution, samples were incubated overnight at 4°C. PBS was used as the negative control. The specimens were rinsed in PBS three times and incubated with the secondary antibody at 37°C for 45 min. Subsequently, the specimens were rinsed again in PBS, developed for 5-10 min, and stained using diaminobenzidine (DAB) (Kit-0016, Fuzhou Maixin Biotechnology Development Co. Ltd., Fuzhou, Fujian Province, China). The specimens were washed under running water, stained with hematoxylin for 5 min, diluted with hydrochloric acid for 30 s, and washed for 5 min. Next, the specimens were dehydrated, cleared, mounted and viewed under an inverted microscope.

RETRACTED

IHC scoring: The IHC results were evaluated by two senior pathologists using a double-blind method. Cells containing yellow to brown cytoplasm or membrane were regarded as positive. Specimens were scored according to the positive-cell rate as follows: positive cells ≤ 5%, 0 point; 6-25% positive cells, 1 point; 26-50% positive cells, 2 points; positive cells > 50%, 3 points. Specimens were also scored based on the staining intensity as follows: negative, 0 points; pale yellow, 1 point; medium yellow, 2 points; pale brown, 3 points. Protein expression was determined using positive-cell rate and staining intensity. The product of positive-cell rate and staining intensity ≥ 3 indicated high expression, and < 3 indicated low expression.

### Cell culture

Cell lines EJ, 5637, T24, and RT-4 were purchased from the Institute of Shanghai Biochemistry and Cell Biology and Chinese Academy of Sciences (Shanghai, China). The cell lines were maintained in a Dulbecco's minimum essential medium (DMEM) (Gibco, Grand Island, New York, USA) with 10% fetal bovine serum (FBS, Purpleflower Holly Leaf; Hangzhou, China) and 1% double antibiotics (100 U/ L penicillin and 100 mg/L streptomycin; Gibco, Grand Island, New York, USA). The cells were incubated at 37°C in a humidified incubator containing 5% CO_2_ in air. After incubation, the cells were detached from the culture surface using 0.25% trypsin (Gibco Company, Grand Island, NY, USA) and then re-plated and cultured for subsequent experiments.

### Cell grouping and transfection

5637 BC cells were divided into control, siRNA-NC (non-specific siRNA with scramble), si-CUL4B (silencing CUL4B), CUL4B (CUL4B overexpression vectors, PLOC-CUL4B purchased from Invitrogen, CA, USA), WIF-1 (100ng/ml, an inhibitor of the Wnt/β-catenin signaling pathway, Sigma-Aldrich Chemical Company, St Louis, Missouri, USA) and CUL4B + WIF-1 groups (transfected with CUL4B and WIF-1) depending on the vector used for transfection. The siRNA sequences were synthesized using GenePharma (Shanghai, China) as follows: siRNA-NC: 5’-UUCUCCGAACGUGUCACGUTT-3’, siRNA-CUL4B: 5’-CCACCCAGAAGUCAUUAAUTT-3’. The 5637 cells or 5637-EGFP cells showing a stable expression of EGFP were used for establishing nude mouse metastatic models of BC in the logarithmic growth phase, which were plated and then transferred into an antibiotic-free medium 24 h later. The medium was replaced with serum-free Opti-MEM once cell density reached a rate of 40-60%. The transfection was conducted after mixing transfection reagents and plasmids or vectors (200 μl) at a cell density of 70% according to the instructions of Lipofectamine 2000 (11668-027, Invitrogen Inc., Carlsbad, California, USA). The samples were cultured at 37°C with 5% CO_2_ for 6 h and upon completion, the medium was replaced with the normal medium containing serum.

RETRACTED

### Quantitative real-time polymerase chain reaction (qRT-PCR)

Total RNA was extracted based on the Trizol method in order to determine the concentration and purity of RNA. According to the instructions of the reverse transcription kit (DRR047S; TAKARA Biotechnology Ltd., Dalian, Liaoning Province, China), 10 μl cDNA was created and 65 μl diethyl pyrocarbonate (DEPC) was added to cDNA for dilution. The qRT-PCR reaction system was as follows: 5 μl SsoFast EvaGreen Supermix (1708882; BIO-RAD, Laboratories, Inc., Hercules, California, USA), 0.5 μl forward primer (10 μM), 0.5 μl reverse primer (10 μM), and 4 μl cDNA. The PCR amplification conditions were as follows: pre-denaturation for 1 min at 95°C, denaturation for 30 s at 95°C, annealing for 5 s at 58°C, and finally extension for 5 s at 72°C with 30 cycles. The primers were synthesized by China Gene Company Limited (Supplementary Table 1). Using glyceraldehyde phosphate dehydrogenase (GAPDH) as the internal reference, each gene was tested three times in each sample. The cycle threshold (CT) value of each reaction was recorded, and the relative expression of the target gene was calculated using the 2^-ΔΔCt^ method [33]. ΔCt= CT (target gene) – CT (internal reference), ΔΔCt = ^ΔΔ^Ct (experiment group) – ^Δ^Ct (control group). The experiment was repeated three times.

### Western blotting

The total protein was extracted from cultured cells of each group. The protein concentration was measured using a bicinchoninic acid (BCA) assay kit and adjusted to the same protein concentration in all groups. Subsequently, 5 × sodium dodecyl sulfate (SDS) loading buffer was added, and protein denaturation was performed at 95°C for 5 min. The samples were electrophoresed using a sodium dodecyl sulfate-polyacrylamide gel electrophoresis (SDS-PAGE), transferred to a membrane and blocked using 5% skim milk overnight. After washing the membrane with tris-buffered saline + Tween-20 (TBST), primary antibodies were added to the samples and incubated at 4°C overnight. The primary antibodies used in the experiment were as follows: cyclinD1 (#2978; diluted at a ratio of 1: 1000; CST, Beverly, Massachusetts, USA), β-catenin (#9587s; diluted at a ratio of 1: 1000; CST, Beverly, Massachusetts, USA), t-GSK3β (ab32391; diluted at a ratio of 1: 1000; Abcam, Inc., Cambridge, Massachusetts, USA), p-GSK3β (ab75814; diluted at a ratio of 1: 1000; Abcam, Inc., Cambridge, Massachusetts, USA), c-myc (ab32072; diluted at a ratio of 1: 1000; Abcam, Inc., Cambridge, Massachusetts, USA), MMP7 (ab207299; diluted at a ratio of 1: 1000; Abcam, Inc., Cambridge, Massachusetts, USA), E-cadherin (#3195; diluted at a ratio of 1: 1000; CST, Beverly, Massachusetts, USA), N-cadherin (#8480; diluted at a ratio of 1: 1000; CST, Beverly, Massachusetts, USA), Vimentin (#5741; diluted at a ratio of 1: 1000; CST, Beverly, Massachusetts, USA), ZEB1 (#ab203829, diluted at a ratio of 1: 1000, Abcam, Inc., Cambridge, Massachusetts, USA), ZEB2 (#ab138222, diluted at a ratio of 1: 500, Abcam, Inc., Cambridge, Massachusetts, USA), Snail1 (#ab180714, diluted at a ratio of 1: 500, Abcam, Inc., Cambridge, Massachusetts, USA), GAPDH (#5174; diluted at a ratio of 1: 1000; CST, Beverly, Massachusetts, USA), and β-actin (ab3280; diluted at a ratio of 1: 1000; Abcam, Inc., Cambridge, Massachusetts, USA). Subsequently, the samples were rinsed in TBST supplemented with a horseradish peroxidase (HRP)-conjugated secondary antibody and cultured for 1 h at 37°C. After rinsing the membrane in TBST, enhanced chemiluminescence (ECL) was employed in order to develop HRP, and HRP was recorded using scanning. The gray value of the target band was analyzed using the ImageJ software. The experiment was repeated three times independently.

RETRACTED

### 3-(4,5-dimethyl-2-thiazolyl)-2,5-diphenyl-2-H-tetrazolium bromide (MTT) assay

The transfected cells were diluted to a specific concentration and plated in a 96-well plate with 5 × 10^3^ cells in each well. The cells were cultured in a 37°C 5%CO_2_ incubator for 24 h, 48 h, and 72 h. Subsequently, 10 μl MTT (Sigma-Aldrich Chemical Company, St Louis, Missouri, USA) was added to the wells in dark conditions. Cells were consequently cultured for 4 h. After draining the nutrient fluid, 100 μl dimethyl sulfoxide (DMSO, Sigma-Aldrich Chemical Company, St Louis, Missouri, USA) was added to the wells in dark conditions. The cells were lysed on an oscillator for 15 min and monitored using a microplate reader (Biotek, Winooski, VT, USA). The optical density (OD) was detected at a wavelength of 570 nm. The experiment was repeated three times independently.

### Transwell assay

After the 3rd generation of cells reaching 80% confluence were cultured in serum-free DMEM for 24 h. The serum-free DMEM was added into the lower Transwell chamber (Corning Inc., Corning, New York, USA) and incubated at 37°C for 1 h. Next, the cells were re-suspended in serum-free DMEM after digestion, counting, and dilution to the concentration of 3 × 10^5^ cells/ml. Then, 100 μl cells were added into the upper chamber, and 600 μl DMEM with 10% serum was added into the lower chamber (serum as a chemotactic factor). Following the Transwell chamber instructions, the cells were incubated for 24 h. Cells in the upper chamber were removed and rinsed in PBS. The cells were then placed in pre-cooled methanol for 30 min, fixed and transferred to the lower chamber. The cells were stained using 0.1% crystal violet solution for 10 min. Six visual fields of the cells were selected, and the cells were photographed and counted using an inverted microscope (Olympus Optical Co., Ltd., Tokyo, Japan). The experiment was repeated three times independently. Matrigel was taken out from a -20°C refrigerator and melted in a 4°C refrigerator for the cell invasion assay. Serum-free DMEM was prepared at a dilution ratio of 1: 10. The cell density was adjusted to the concentration of 1.0 × 10^5^ cells/ml. Subsequent steps were taken following similar procedure as cell migration. The experiment was repeated three times independently.

RETRACTED

### Xenograft model in nude mice

A total of 32 BALB/c nude mice (age, 5-8 weeks; weight, 18-20 g) purchased from the Animal Center of Sun Yat-sen University (Guangzhou, China) were assigned to the control, siRNA-NC, si-CUL4B, and CUL4B groups for transfection, with 8 mice in each group. The nude mice were fed a normal diet and maintained at a constant temperature, and the mice were observed for a week prior to tumor inoculation. The transfected cells were digested, centrifuged at a rate of 1000 rpm for 5 min, and rinsed in PBS. The cells were then collected and mixed with diluted Matrigel at a high concentration (PBS: Matrigel = 2: 1). Subcutaneous injections were used in order to inoculate the nude mice with 5 × 10^6^ tumor cells. Weight of the nude mice was recorded every 5 days. The long and short axis diameters of the tumors were recorded using a venire caliper. The transfected mice were sacrificed by cervical dislocation 35 days after inoculation. Consequently, the tumors were weighed and recorded. Gross tumor volume (mm^3^) was calculated using the formula: ½ × (L × W^2^) (L is long axis diameter and W is short axis diameter). At the 15^th^ day after inoculation, 3 mice in each group were sacrificed by cervical dislocation. The tumor tissues were separated and fixed with 4% paraformaldehyde. QRT-PCR and IHC were employed in order to detect the mRNA and protein expression of EMT markers.

### Nude mouse metastatic models of BC by tail vein injection

A total of 32 BALB/c nude mice (age, 5-8 weeks; weight, 18-20 g) purchased from the Animal Center of Sun Yat-sen University (Guangzhou, China) were assigned to the control, siRNA-NC, si-CUL4B and CUL4B groups, with 8 mice in each group. The nude mice were fed a normal diet and maintained at a constant temperature, and the mice were observed for a week prior to tumor inoculation. The transfected cells were digested, centrifuged at a rate of 1000 rpm for 5 min, and rinsed in PBS. The cells were then collected and mixed with diluted Matrigel (PBS: Matrigel = 2: 1). After rinsing the tails of the nude mice in hot water at 50°C for 3-5 min to dilate the blood vessels, a cell suspension (0.2 ml) was injected into the mice via the tail vein. After successful injection, the mice were maintained in clean cages for observing hematogenous metastasis using a LT-9MACIMSYSPULS fluorescence microscope. In order to observe lung metastases, the mice were sacrificed and dissected 2 months after inoculation.

RETRACTED

### Statistical analysis

Statistical analyses were performed using the SPSS21.0 software (SPSS Inc., Chicago, Illinois, USA). The experiments were repeated at least three times. Measurement data were presented as mean ± standard deviation (SD). If the recorded data were normally distributed and had homogeneous variance, t-tests were used for comparisons between two groups and one-way analysis of variance (ANOVA) was used for comparisons among multiple groups, The Wilcoxon rank sum test was performed if the recorded data were abnormally distributed and had inhomogeneous variance. Enumeration data were expressed as percentages. *P* < 0.05 was considered statistically significant.

## SUPPLEMENTARY MATERIALS TABLE



## References

[1] Bansal N, Gupta AK, Gupta A, Sankhwar SN, Mahdi AA (2016). Serum-based protein biomarkers of bladder cancer: a pre- and post-operative evaluation. J Pharm Biomed Anal.

[2] Wang J, Zhang X, Wang L, Dong Z, Du L, Yang Y, Guo Y, Wang C (2015). Downregulation of urinary cell-free microRNA-214 as a diagnostic and prognostic biomarker in bladder cancer. J Surg Oncol.

[3] Freedman ND, Silverman DT, Hollenbeck AR, Schatzkin A, Abnet CC (2011). Association between smoking and risk of bladder cancer among men and women. JAMA.

[4] Witjes JA, Comperat E, Cowan NC, De Santis M, Gakis G, Lebret T, Ribal MJ, Van der Heijden AG, A; Sherif, European Association of Urology (2014). EAU guidelines on muscle-invasive and metastatic bladder cancer: summary of the 2013 guidelines. Eur Urol.

[5] Babjuk M, Oosterlinck W, Sylvester R, Kaasinen E, Bohle A, Palou-Redorta J, Roupret M, European Association of Urology (2011). EAU guidelines on non-muscle-invasive urothelial carcinoma of the bladder, the 2011 update. Eur Urol.

RETRACTED

[6] Gregg JR, Cookson MS, Phillips S, Salem S, Chang SS, Clark PE, Davis R, Stimson CJ, Aghazadeh M, Smith JA, Barocas DA (2011). Effect of preoperative nutritional deficiency on mortality after radical cystectomy for bladder cancer. J Urol.

[7] Arfaoui AT, Mejri S, Belhaj R, Karkni W, Chebil M, Rammeh S (2016). Prognostic value of immunohistochemical expression profile of epidermal growth factor receptor in urothelial bladder cancer. J Immunoassay Immunochem.

[8] Raj GV, Karavadia S, Schlomer B, Arriaga Y, Lotan Y, Sagalowsky A, Frenkel E (2011). Contemporary use of perioperative cisplatin-based chemotherapy in patients with muscle-invasive bladder cancer. Cancer.

[9] TR; Griffiths (2013). Action on Bladder Cancer. Current perspectives in bladder cancer management. Int J Clin Pract.

[10] He F, Lu D, Jiang B, Wang Y, Liu Q, Liu Q, Shao C, Li X, Gong Y (2013). X-linked intellectual disability gene CUL4B targets Jab1/CSN5 for degradation and regulates bone morphogenetic protein signaling. Biochim Biophys Acta.

[11] Wang X, Chen Z (2016). Knockdown of CUL4B suppresses the proliferation and invasion in non-small cell lung cancer cells. Oncol Res.

[12] Song B, Zhan H, Bian Q, Li J (2015). Knockdown of CUL4B inhibits proliferation and promotes apoptosis of colorectal cancer cells through suppressing the Wnt/beta-catenin signaling pathway. Int J Clin Exp Pathol.

[13] Jiang T, Tang HM, Wu ZH, Chen J, Lu S, Zhou CZ, Yan DW, Peng ZH (2013). Cullin 4B is a novel prognostic marker that correlates with colon cancer progression and pathogenesis. Med Oncol.

[14] Chen Z, Shen BL, Fu QG, Wang F, Tang YX, Hou CL, Chen L (2014). CUL4B promotes proliferation and inhibits apoptosis of human osteosarcoma cells. Oncol Rep.

[15] Iwai S, Yonekawa A, Harada C, Hamada M, Katagiri W, Nakazawa M, Yura Y (2010). Involvement of the Wnt-beta-catenin pathway in invasion and migration of oral squamous carcinoma cells. Int J Oncol.

[16] Kim SS, Cho HJ, Lee HY, Park JH, Noh CK, Shin SJ, Lee KM, Yoo BM, Lee KJ, Cho SW, Cheong JY (2016). Genetic polymorphisms in the Wnt/beta-catenin pathway genes as predictors of tumor development and survival in patients with hepatitis B virus-associated hepatocellular carcinoma. Clin Biochem.

[17] van Loosdregt J, Fleskens V, Tiemessen MM, Mokry M, van Boxtel R, Meerding J, Pals CE, Kurek D, Baert MR, Delemarre EM, Grone A, Koerkamp MJ, Sijts AJ (2013). Canonical Wnt signaling negatively modulates regulatory T cell function. Immunity.

[18] Capietto AH, Kim S, Sanford DE, Linehan DC, Hikida M, Kumosaki T, Novack DV, Faccio R (2013). Down-regulation of PLCgamma2-beta-catenin pathway promotes activation and expansion of myeloid-derived suppressor cells in cancer. J Exp Med.

RETRACTED

[19] Cai J, Guan H, Fang L, Yang Y, Zhu X, Yuan J, Wu J, Li M (2013). MicroRNA-374a activates Wnt/beta-catenin signaling to promote breast cancer metastasis. J Clin Invest.

[20] Qian Y, Yuan J, Hu H, Yang Q, Li J, Zhang S, Jiang B, Shao C, Gong Y (2015). The CUL4B/AKT/beta-catenin axis restricts the accumulation of myeloid-derived suppressor cells to prohibit the establishment of a tumor-permissive microenvironment. Cancer Res.

[21] Li L, Li W (2015). Epithelial-mesenchymal transition in human cancer: comprehensive reprogramming of metabolism, epigenetics, and differentiation. Pharmacol Ther.

[22] Malik S, Villanova L, Tanaka S, Aonuma M, Roy N, Berber E, Pollack JR, Michishita-Kioi E, Chua KF (2015). SIRT7 inactivation reverses metastatic phenotypes in epithelial and mesenchymal tumors. Sci Rep.

[23] Kotiyal S, Bhattacharya S (2014). Breast cancer stem cells, EMT and therapeutic targets. Biochem Biophys Res Commun.

[24] Schindl M, Gnant M, Schoppmann SF, Horvat R, Birner P (2007). Overexpression of the human homologue for Caenorhabditis elegans cul-4 gene is associated with poor outcome in node-negative breast cancer. Anticancer Res.

[25] Yuan J, Han B, Hu H, Qian Y, Liu Z, Wei Z, Liang X, Jiang B, Shao C, Gong Y (2015). CUL4B activates Wnt/beta-catenin signalling in hepatocellular carcinoma by repressing Wnt antagonists. J Pathol.

[26] Cheng AS, Lau SS, Chen Y, Kondo Y, Li MS, Feng H, Ching AK, Cheung KF, Wong HK, Tong JH, Jin H, Choy KW, Yu J (2011). EZH2-mediated concordant repression of Wnt antagonists promotes beta-catenin-dependent hepatocarcinogenesis. Cancer Res.

[27] Tomita K, van Bokhoven A, van Leenders GJ, Ruijter ET, Jansen CF, Bussemakers MJ, Schalken JA (2000). Cadherin switching in human prostate cancer progression. Cancer Res.

[28] Nakajima S, Doi R, Toyoda E, Tsuji S, Wada M, Koizumi M, Tulachan SS, Ito D, Kami K, Mori T, Kawaguchi Y, Fujimoto K, Hosotani R, Imamura M (2004). N-cadherin expression and epithelial-mesenchymal transition in pancreatic carcinoma. Clin Cancer Res.

[29] Yuan J, Jiang B, Zhang A, Qian Y, Tan H, Gao J, Shao C, Gong Y (2015). Accelerated hepatocellular carcinoma development in CUL4B transgenic mice. Oncotarget.

[30] Fu J, Lv X, Lin H, Wu L, Wang R, Zhou Z, Zhang B, Wang YL, Tsang BK, Zhu C, Wang H (2010). Ubiquitin ligase cullin 7 induces epithelial-mesenchymal transition in human choriocarcinoma cells. J Biol Chem.

[31] Dong J, Wang XQ, Yao JJ, Li G, Li XG (2015). Decreased CUL4B expression inhibits malignant proliferation of glioma in vitro and in vivo. Eur Rev Med Pharmacol Sci.

[32] Shparyk Ia V (1998). [New classification of malignant tumors TNM (5th edition)]. [Article in Ukrainian]. Klin Khir.

RETRACTED

[33] Tuo YL, Li XM, Luo J (2015). Long noncoding RNA UCA1 modulates breast cancer cell growth and apoptosis through decreasing tumor suppressive miR-143. Eur Rev Med Pharmacol Sci.

